# Analysis of the Effectiveness of Nursing Interventions in Critically Ill Patients in Respiratory Medicine

**DOI:** 10.1155/2022/1193282

**Published:** 2022-01-25

**Authors:** Li-jing Wu, Wen-wen Jiao, Huan-huan Wang, Guo Li, Ping Li, Shun-jing Wang

**Affiliations:** ^1^Nursing Department, Dongying Traditional Chinese Medical Hospital, Beier Road 107, Development Zone, Dongying, Shandong, China; ^2^Department of Respiratory and Gastroenterology, Dongying Traditional Chinese Medical Hospital, Beier Road 107, Development Zone, Dongying, Shandong, China; ^3^Department of Critical Care Medicine, Dongying Traditional Chinese Medical Hospital, Beier Road 107, Development Zone, Dongying, Shandong, China

## Abstract

**Objective:**

To enhance and analyze the clinical effectiveness of implementing quality nursing interventions in the clinical care of critically ill patients in respiratory medicine.

**Methods:**

Clinical data of respiratory medicine patients treated in our hospital over the years were collected and 96 patients who met the requirements of the purpose of this study and the sample inclusion criteria were selected as the study subjects from the patients treated between April 2019 and January 2020. According to the care methods received by the patients in our hospital, 48 of them who implemented conventional care were used as the control group, and another 48 patients who were given quality care interventions were used as the observation group. The data were statistically recorded and comparatively analyzed for the indicators such as nursing oxygen index, heart rate, and clinical treatment efficiency of patients in both groups.

**Results:**

Compared with the control group, patients in the observation group who received quality nursing intervention had more significant improvement in blood oxygen index and heart rate after nursing care; the clinical treatment efficiency of patients in the observation group was significantly higher than that of the control group (95.83% vs. 81.25%). The data comparison between the groups showed a significant difference, *P* < 0.05, which was statistically significant.

**Conclusion:**

Adding quality nursing interventions to the implementation of conventional care for patients with respiratory diseases can better improve patients' clinical symptoms, accelerate their clinical recovery, improve and enhance prognosis, and further improve clinical outcomes.

## 1. Introduction

Since the outbreak in December 2019, severe acute respiratory syndrome coronavirus 2 (SARS-CoV-2) has infected more than 151 million people worldwide. More than 3.1 million people died from the 2019 coronavirus disease (COVID-19), which is caused by SARS-CoV-2. The virus mainly affects the upper respiratory tract and lungs, causing pneumonia of varying severity. In addition, through direct and indirect pathogenesis, SARS-CoV-2 may cause a variety of extrapulmonary and vascular manifestations [1]. Since 2021, new variants of the new coronavirus severe acute respiratory syndrome have emerged rapidly, from an outbreak to a global pandemic [1]. The global incidence of respiratory diseases and complications is increasing. Therefore, new treatment and prevention methods need to be studied [2]. There was also a life-saving strategy to solve acute respiratory distress syndrome. The method was to ventilate the critically ill patients in the prone position, but it would bring adverse consequences such as skin damage [3].

Respiratory infections spread quickly, and doctors will advise you to use masks or respirators, keep your hands clean, and keep your distance from others to limit the transmission of these diseases. [4]. We thought of implementing high-quality nursing interventions to provide better services to critically ill patients in the Department of Respiratory Medicine. High-quality care can better improve the clinical symptoms of patients and speed up the clinical recovery of patients, but poor quality of care includes reduced availability and accessibility of services and limited participation in health promotion and can also lead to the hospitalization of adults with developmental disabilities. The rate and complication rate are higher [5]. In general, the review emphasized that inequities in healthcare can be decreased through quality care initiatives. Incorporating clinical nursing and clinical experience with critically ill patients in internal medicine into nursing education will reduce inequity in this service, enhance and increase prognosis, and improve the clinical treatment effect even more.

## 2. Methods

### 2.1. General Information

Ninety-six patients with severe respiratory disease admitted from April 2019 to January 2020 were selected and randomly divided into control and observation groups, with 48 cases in each group. The baseline of each group is exhibited in Table 1. In the control group, there were 26 male patients and 22 female patients, aged 44–78 years, with a mean age of 65.2 ± 3.5 years; in the observation group, there were 28 male patients and 20 female patients, aged 45–79 years, with a mean age of 65.3 ± 3.4 years. There was no significant difference between the two groups when comparing gender and age (*P* > 0.05). Inclusion criteria: meeting the diagnostic criteria for respiratory diseases, meeting the criteria for determining serious respiratory diseases, informed consent of patients or family members for this study, and approval of the medical ethics committee. Exclusion criteria: patients with combined malignancy, patients with other important organ diseases such as the heart, liver, and kidney, patients with cognitive or communication disorders, and patients with incomplete clinical information. The control group took routine nursing interventions in respiratory medicine including medication care and diet care, while following the medical advice to carry out routine condition observation care.

### 2.2. Experimental Groupings

In the observation group, comprehensive quality nursing interventions were provided on the basis of conventional nursing care. Psychological nursing was carried out to establish close communication with patients for their anxiety and depression due to disease factors and to carry out effective psychological interventions, understand patients' inner concerns, answer their questions, and correct misconceptions. We help patients adopt effective methods to relieve their emotions, maintain a good state of mind, and actively cooperate with nursing care. All vital signs were closely monitored and effective measures were taken to intervene and prevent various adverse symptoms that may occur. At any time, the patient's heart rate, respiratory rate, respiratory depth, and other vital signs were monitored and recorded and the patient's health was assessed, and the nursing program was altered as needed. Oxygen therapy care was carried out, and effective oxygen therapy care was taken for respiratory medicine patients with severe respiratory distress, using nasal mask oxygenation to correct the patient's hypoxic state. Aerosol was correctly used; we paid attention to good sterilization treatment to avoid infection. Mechanical ventilation care was given, airway secretions were regularly observed and cleaned, and correct operation was ensured during oxygen inhalation to avoid damage to the mucosa. There should be reasonable wetting of the airway to keep it moist and reduce infection. the indications for deconditioning were strictly grasped; the machine was withdrawn in time and the duration of mechanical ventilation was shortened.

### 2.3. Evaluation Indicators

Heart rate and respiratory rate levels, as well as blood oxygen index levels, were compared between the two groups before and after care.

### 2.4. Mitigation Measures

If the patient is in remission, the patient should be encouraged to live a healthy lifestyle, cease smoking and drinking, avoid airway infections, and wear suitable clothes when the weather changes to avoid becoming cold. At the same time, the patient should be rehabilitated according to his or her recovery status to ensure that he or she maintains a clear airway.

### 2.5. Statistical Analysis

SPSS 20.0 software was used to process the data. The measurement data were expressed as mean ± standard deviation. *T*-test and Wilcoxon rank test was used, and *P* < 0.05 was considered a statistically significant difference.

## 3. Experimental Results

### 3.1. Comparison of Heart Rate and Respiratory Rate between the Two Groups before and after Care

Before care, there was no significant difference in heart rate and respiratory rate between the two groups (*P* > 0.05); after care, the heart rate (80.25 ± 8.41 beats/min) and respiratory rate (22.05 3.21 beats/min) in the observation group were better than the control group; there was a significant difference (*P* < 0.05) (Tables 2∼3).

### 3.2. Comparison of Blood Gas Index Levels before and after Care between the Two Groups

Before care, there was no significant difference in blood gas index levels between the two groups compared to each other (*P* > 0.05); after care, observation group was with PaO_2_ (74.05 ± 7.14 mmHg) and PaCO_2_ (65.49 ± 6.08 mmHg), which were better than the control group. There was a significant difference (*P* < 0.05) (Tables 4∼5).

### 3.3. Comparison of Treatment Efficiency between Two Groups of Patients

Statistical analysis of the efficacy of all patients participating in this study showed that only two patients in the observation group had no significant changes in relevant clinical symptoms and performance after care, and their total clinical treatment efficiency reached 95.83% (46/48), which was significantly higher than that of the control group (81.25%, 39/48). *P* < 0.05, the difference was statistically significant (Table 6).

## 4. Discussion

Since China reported its first case at the end of 2019, the coronavirus disease (COVID-19) has spread rapidly in various countries and regions, leaving devastating traces on its transmission path, everywhere. COVID-19 is mainly a respiratory disease that mainly affects the lungs; the involvement of other organs, including the cardiovascular system, has been widely recognized [6].

The unprecedented long-term coronavirus disease 2019 (COVID-19) pandemic has exacerbated the severity of the mental health disaster. During this treatment period, nurses and healthcare providers play a key role in all stages of disaster management. Nurses need to be prepared and capable of responding to such disasters [7]. Unmet care needs and poor quality of care for this resident population have been widely reported [1].

In our study, first, we split the patients into two groups: control and observation, with both male and female patients. For the control group, we used standard respiratory medicine nursing techniques. This included medication care and dietary care, and at the same time, we carried out measures such as routine condition observation care as prescribed by the doctor, and secondly, for the observation group, we adopted comprehensive quality care interventions on the basis of routine care and recorded their heart rate, respiratory rate, respiratory depth, and other vital signs at any time and compared them. Finally, through data analysis, we found that the total clinical treatment efficiency of patients with quality nursing intervention was significantly higher than that of the control group, and the quality nursing intervention was positively correlated with the response rate of patients' conditions.

However, high-quality care also requires many areas of improvement, including healthcare improvement training and certification; healthcare improvement project activities; healthcare improvement counseling, teaching, and curriculum activities; and healthcare improvement honors, awards, and recognition. This combination fosters nurses' professional esteem as well as their input and effect on healthcare improvement, and it encompasses the full range of cross-professional healthcare improvement. [5]. In addition, leaders play a vital role in the quality of care in nursing homes or hospitals. However, few studies have explored the views of senior management on how to ensure that residents receive high-quality care. This is also one of our future research directions to improve the quality of care [8]. Moreover, Our trial sample is still small and has limitations for experimental analysis, and we will expand the study in the future to provide better support for nursing interventions.

## 5. Conclusion

By carrying out quality care in respiratory medicine, we can effectively improve the quality of care, promote a good relationship with respiratory intensive care patients, improve patient satisfaction, and have a good thought on clinical treatment and service experience, and our study is worth promoting.

## Figures and Tables

**Table 1:** Baseline.

	Control group	Observation group	*P* value
Gender			>0.05
Male	26	28	
Female	22	20	
Age			>0.05
	65.2 ± 3.5	65.3 ± 3.4	

**Table 2:** Heart rate comparison.

Group	HR (heart rate/min)	
	Before	After
Control (*n* = 48)	105.62 ± 12.78	86.74 ± 9.63
Observation (*n* = 48)	104.31 ± 12.61	80.25 ± 8.41
*t* value	0.40	2.78
*P* value	0.69	0.01

**Table 3:** Respiratory rate comparison.

Group	RR (respiratory rate/min)	
	Before	After
Control (*n* = 48)	29.63 ± 4.82	25.42 ± 3.97
Observation (*n* = 48)	29.57 ± 4.83	22.05 ± 3.21
*t* value	0.05	3.62
*P* value	0.96	<0.01

**Table 4:** PaO_2_ comparison.

Group	PaO_2_ (mmHg)	
	Before	After
Control (*n* = 48)	52.36 ± 5.48	68.49 ± 6.37
Observation (*n* = 48)	51.79 ± 5.40	74.05 ± 7.14
*t* value	0.41	3.18
*P* value	0.69	<0.01

**Table 5:** PaCO_2_ comparison.

Group	PaCO_2_ (mmHg)	
	Before	After
Control (*n* = 48)	81.58 ± 8.97	70.12 ± 7.65
Observation (*n* = 48)	82.36 ± 9.02	65.49 ± 6.08
*t* value	0.34	2.60
*P* value	0.73	0.01

**Table 6:** Total effective rate of nursing.

Group	Ineffective	Effective	Conspicuous effect	After
Control (*n* = 48)	9 (18.75)	22 (45.83)	17 (35.41)	39 (81.25)
Observation (*n* = 48)	2 (4.17)	21 (43.75)	25 (52.08)	46 (95.83)
*Z*	0.344	—	—	2.595
*P* value	0.732	—	—	0.012

## Data Availability

The datasets used and analyzed during the current study are available from the corresponding author on reasonable request.
